# Design and Research of Remote Monitoring System for Sports Injury Rehabilitation Training

This article has been retracted.

**DOI:** 10.1155/2021/4390089

**Published:** 2021-09-27

**Authors:** Hongyan Liu, Panlong Qin, Ruiming Qi

**Affiliations:** Department of Physical Education, Hebei Academy of Fine Arts, Hebei 050700, China

## Abstract

In order to study the sports injuries that often occur in athletes' training and competition and solve the problems of low monitoring accuracy of injury mode data and large difference of resistance signal waveforms in the traditional monitoring system, this paper proposes the application of wireless sensor network in monitoring process. The accuracy of data monitoring with 9 different degree injury modes set by 1–9 squares in the traditional system is lower, while the accuracy of sports injury rehabilitation monitoring based on wireless sensor network is higher, which can be maintained above 90%. The experimental results show that the monitoring system has high monitoring accuracy of damage mode data and small difference of resistance signal waveform. It is basically consistent with the actual waveform.

## 1. Introduction

Sports injuries refer to various injuries that occur during the process of sports training. The injured parts are directly related to the sports training received by athletes themselves. For example, for gymnasts, the injured parts are shoulder, waist, or wrist. This is mainly because gymnasts often practice supporting, jumping and somersault, and other related techniques. The injuries of tennis players and javelin throwers mostly occur in elbow. To a great extent, the causes of athletes' sports injuries are caused by insufficient training level, inaccurate movements, and lack of protection awareness [1]. Before sports, there are not enough preparations for activities, poor physical fitness, inability to adapt to the surrounding environment, and improper competition organization. However, at present, the arrangement of rehabilitation for athletes' sports injuries is largely based on the advice of team doctors and the way of rehabilitation training [2]. This paper proposes the application of wireless sensing network in the monitoring process. The rehabilitation robot is equipment that assists patients in rehabilitation training as a new rehabilitation training platform.

## 2. Literature Review

The rehabilitation robot developed in this paper, which combines information technology, intelligent control technology, and entity-based mechanical structure, is equipment that can assist patients in rehabilitation training. As a new type of the rehabilitation training platform, the robot is an effective clinical intervention means to assist physicians in the reconstruction of patients' motor function. With the upper limb rehabilitation training system developed by Capecci et al., as the representative [3], the early sports rehabilitation robot provided resistance and driving force through the spring support of free inertia balance, which was simple in the design and could only assist patients in rehabilitation training to a limited extent. Until 1980s, with the deepening of relevant scientific research, some rehabilitation robots with reliable performance appeared in the international community [4]. For example, Khan's rehabilitation robot, researched and developed by Zurich University in Switzerland, embeds the training mode of predetermined trajectory mode, and the attending physician first guides the patient's limbs to move, the system records the patient's motion trajectory, and then the robot reproduces these trajectories [5]. After setting different repetition speeds and frequencies, patients can choose different training levels according to their own state and complete the rehabilitation training process according to the robot's guidance and follow the trajectory. The platform also has a “point arrival” mode of guiding the motion trajectory to reach the point through the image. And, the “guiding force support” mode, which assists in supporting the patient's training action, determines the training track by the patient, and simulates the training parameters by the system, provides a new idea for the rehabilitation robot product to transition from a single resistance or support mode to a multitraining mode. There are also some typical training robot products. The patient's spatial motion range and state are optimized, and a relatively perfect man-machine interaction control system is designed, which can stimulate the patient's training activities from hearing, vision, and other senses [6]. The typical one is Armeo series rehabilitation robots developed by Hocoma Company of Switzerland. And, a new multi-degree-of-freedom upper limb rehabilitation training robot is developed by University of Shanghai for Science and Technology [7]. Aiming at the young people with dyskinesia, Huang Junda et al. designed and developed a set of somatosensory rehabilitation training system, Kinerehab, which is specially used to increase patients' rehabilitation enthusiasm and improve the efficiency of rehabilitation activities. By detecting and recording the actions of subjects, we match the acquired patient joint position information with the existing database in the system, judge the degree of coincidence between the patient and the standard action, and then calculate the accuracy of the action in place. The system has a relatively friendly man-machine interaction interface, which can reflect the rehabilitation effect of patients on the screen in the form of animation, so as to facilitate intervention and guidance for patients [8]. It can also increase their interest and patience. In the process of rehabilitation training, the system will automatically record the training status of the subjects, so as to help doctors quickly check the progress and decide the follow-up rehabilitation content and progress. The Kinerehab system can significantly improve the muscle endurance of patients with dyskinesia and help them deal with some daily tasks alone. Shen et al. focused on repetitive training methods for patients with nervous system damage or pathological changes and developed a set of sports rehabilitation system specially used for training the balance ability of patients with nervous system damage [9]. On the basis of extracting the depth sensing information captured by the equipment, the system reconstructs the three-dimensional model of human body-virtual human and introduces the virtual scene into the development platform, so as to carry out balanced rehabilitation training for patients in the form of simple games. In the course of the game, the system uses the camera to get the image information in real time and uses the virtual human to reflect the tracking results of the sensor. The subjects, after receiving the feedback prompt information sent by the system, can correct the balance posture of one's shoulder, elbow, and other parts. And, by doing interactive training with virtual human, we can enhance our sense of balance. Similarly, the system patients' scores in each game stage will be automatically recorded, and rehabilitation results will be accepted [10].

In view of the above problems, this paper proposes a sports injury rehabilitation monitoring system based on wireless sensor network. Because the network nodes have local processing capability, the running speed and flexible state of the system can be improved by serially processing all lines of the traditional system and making centralized decisions. It can be seen from the experimental verification results that the system has high accuracy in sports injury rehabilitation monitoring. The waveform of resistance signal is basically consistent with the actual waveform, and the monitoring effect is good.

## 3. Research Methods

### 3.1. Principles of System Development

(1) The principle of advancement: the choice of system hardware must choose the current computer hardware, so as to ensure that the system can adapt to the growing business needs of the system. On the software side, the latest database technology and system architecture design are selected. (2) Safety and reliability: the information management system contains a lot of personal information of athletes and coaches. Therefore, strengthening the data security of information management system has become its primary goal. Secondly, ensuring the reliable operation of the system is also one of the important principles of the system design. By enhancing the compatibility between hardware and software, the operation of the system can be guaranteed. (3) Scalability: the design of the system must have a certain sense of advancement, in order to ensure that the system will be advanced in the future. At the same time, with the development of system business, its requirements are constantly changing, so it is inevitable to expand the original system functions. Reservation of functional interfaces and retention of system extensibility are prerequisites for retaining the advanced nature of the system. (4) Openness and portability: openness means that, in the process of designing the system, the system must meet the open design standards so that different hardware and software must be compatible when designing different indexes, such as database and middleware, which must meet the standards, so as to ensure the reliable operation of the system. (5) In the development of the system, the first consideration is advanced, reliable, and safe, but from an economic point of view, it must also reflect the performance and high cost performance of the product, so as to maximize economic and social benefits. Because the wireless sensor network terminal node is installed on the sports injured person, it takes a long time, so each module is designed according to the principle of chip selection and circuit design with low power consumption and microvolume [11, 12].

### 3.2. IRIS Dataset Module

IRIS dataset module of wireless sensor network terminal integrates processing chip and RF chip and provides data for the controller and the wireless transceiver. At the same time, the IRIS dataset can be used to realize wireless measurement, which is connected with the dataset module through standard extended interface [13, 14]. The specific interface definition is shown in Table 1.

After conditioning the circuit, the data transmission channel module can be simulated by the sensor, and analog conversion can be carried out in the dataset, and all data can be sent by the dataset module. In addition, the front-end circuit for physiological parameters should be provided at the sensor interface to provide power for the whole circuit.

#### 3.2.1. Power Supply Module

Because the wireless sensor module needs to be installed on the injured person, the unit providing power for this purpose is strictly limited. Considering the working time of nodes, the power supply energy is renewable or exists in the form of unit power supply conversion, and two batteries are designed in the circuit to supply power.

#### 3.2.2. ECG Signal Acquisition Module

Electrocardiogram not only contains athletes' physiological state information but also can accurately extract athletes' electrocardiogram, which can be analyzed to evaluate the effect of rehabilitation training [15, 16]. According to that construction of the module, both diastole and contraction are accompanied by the change of electrocardiogram waveform, and the conduction of cardiac potential can bring potential changes to the surface of human body. The value of cardiac activity changes can be recorded from any body surface electrode, and the change of cardiac activity potential can be observed from the curve, and the movement injury condition, heart change, signal transmission, and process of injury rehabilitation can be reflected from the fluctuation point and atrial successive potential changes. The specific ECG waveform diagram is shown in Figure 1.

It can be seen from Figure 1 that the period of the ECG signal includes five waveforms, *A*, *B*, *C*, *D*, and *E*, which, respectively, represent the activity of beating heart. Section *A* reflects the changes of potential and time during depolarization of left and right atria; *B* represents the change from atrial depolarization to ventricular depolarization; *C* represents the change of potential and time during depolarization of left and right ventricles; *D* reflects the potential and time changes in the early stage of ventricular repolarization; *E* reflects the potential changes in late ventricular repolarization. It can be seen from the electrocardiogram that the wave group composed of a series of waveforms represents a beating cycle of the heart, and one wave group includes *A* wave and *BCD* wave group. Clinical diagnosis can be made by analyzing the wave group in electrocardiogram. Because ECG signal is easily interfered by line noise, in order to obtain higher signal-to-noise ratio, low noise components should be selected to reduce noise [17, 18].

### 3.3. Design of System Software

#### 3.3.1. Design of Node Software

Wireless sensor network system is the core part of the whole monitoring system software. The system is responsible for data acquisition and forwarding and receiving functions and is composed of various sensor network node software. Node software design mainly includes the research and development of sensor network hierarchical routing protocol and node software module. Combined with its own characteristics, the design of wireless sensor network hierarchical protocol is as follows. (1) Prolong network life, that is, save energy consumption, prolong network service life, reduce energy consumption, and save energy on the premise of ensuring normal operation [19, 20]. Because the relay node command received by the acquisition point needs to execute specific acquisition function, the system will be in a dormant state, avoiding long-distance transmission, thus saving energy. (2) Synchronize data collection time between different nodes in the software design; data packet parameters are defined to improve the accuracy of data recording. The acquisition point is triggered repeatedly on a timer, and the sending time can be recorded as T1. The specific calculation is as follows:

(1) $$\begin{array}{c} T1=T2*T3, \end{array}$$

where T1 is the sending time, T2 is a parameter, and T3 is the time interval. In the subsequent data processing process, all data packet parameters are read, which can realize the time synchronization function of data collection among different nodes.

#### 3.3.2. Analysis of Operating System

According to the analysis of the operating system structure, an open source micro-operation technology can be adopted, which can be used for framework programming, and a set of necessary components can be connected through the network embedded system framework so that the operating system can be compiled for the development of applications, which is convenient for the implementation of operations between components. The operational structure design applied in that system can be divided into four layers. They are main component, application component, system component, and abstract component.

## 4. Result Analysis

After the hardware structure and software function of the system are designed, in order to realize sports injury rehabilitation monitoring based on wireless sensor network, the system needs to be verified by experiments.

### 4.1. Experimental Results and Analysis of Sports Injury Location

The topology arrangement of wireless sensor network is shown in Figure 2.

In this structure, carbon fiber load material is used as the resistance strain gauge, and four adjacent resistors are used as the vertices of the strain gauge to form a quadrilateral figure. The quadrilateral figure is divided into 9 sizes. The redundant corners are removed, the resistors of 10 channels are used as strain gauges, and the nodes are forwarded at the cluster head, one of which is a relay node. After the strain gauges of resistors are arranged, they are connected with a signal conditioning circuit, and simulated damages are loaded at the centers of the nine squares with the same size, and the signals are transmitted to the wireless sensor network. The network is urged to collect node data in time. After receiving the command, the node began to collect and transmit data, which was repeated for 10 times, thus obtaining 9 groups of experimental data. After data acquisition, the network needs to quantify the learning vector of competitive neural network by using self-organizing learning ability, so as to determine the motion.

The location of injury is convenient for rehabilitation monitoring. During the experiment, the loaded area is taken as the experimental area, in which 1–9 squares are set as 9 different damage modes, and the learning vector quantization neural network is used to identify different damage modes.  Table 2 shows the collected sensing data and mode judgment results.

According to the data collected in Table 2 and the judgment results, the traditional monitoring system is compared with the monitoring system in this paper, and the results are shown in Table 3.

From Table 3, it can be seen that the data monitoring accuracy rate of 9 injury modes with 1–9 squares in the traditional system is lower, while the monitoring accuracy rate of sports injury rehabilitation based on wireless sensor network is higher, which can be maintained above 90%.

### 4.2. Experimental Results and Analysis of Physiological Parameter Monitoring

The monitoring experiment of physiological parameters during exercise includes the collection of ECG, body temperature, and skin resistance, and each module needs to be carefully tested. In this experiment, skin resistance signals were used as experimental data. Because that circuit is relatively simple, qualitative analysis is adopted to determine the relationship between state changes, and after repeated tests, the resistance value in the circuit is adjusted. Thus, an ideal skin resistance signal waveform is obtained, as shown in Figure 3.

According to the skin resistance signal waveform information obtained in Figure 3, the resistance signals monitored by the traditional system and the system in this paper are compared, and the result is shown in Figure 4.

It can be seen from Figure 4 that, after the skin is stimulated, the resistance signal monitored by the traditional system is quite different from the monitoring result in this paper, and the monitoring result in this paper is basically consistent with the actual waveform.

### 4.3. Experimental Conclusion

The emotional recognition based on physiological parameters is used for experimental verification. The comparison results show that the traditional monitoring system has problems such as low monitoring accuracy of damage mode data and large difference of resistance signal waveform. However, the monitoring accuracy of sports injury rehabilitation based on wireless sensor network is higher, and the resistance signal is basically consistent with the actual waveform.

## 5. Conclusion

There is no line constraint in the system of the wireless sensor network system, which greatly increases the monitoring range so that the original monitoring of some areas can only be extended to global monitoring. Distributed monitoring system composed of wireless sensing network can greatly reduce the line connection between components and the difficulty of system construction. In the experimental results, the motion injury recovery monitoring accuracy based on wireless sensing network is high, and the resistance signal is basically consistent with the actual waveform. In the sports injury rehabilitation system, under the condition of athletes' injury rehabilitation management, the significance of building a sports system is to study the recovery training of athletes' injury more comprehensively and scientifically and add a dietary nutrition management module in the system, so as to better promote the recovery training of athletes.

## Figures and Tables

**Figure 1:** Typical ECG waveform.

**Figure 2:** Schematic diagram of topological structure of wireless sensor network.

**Figure 3:** Skin resistance signal waveform.

**Figure 4:** Comparison results of monitoring resistance signals of two systems.

**Table 1:** Sensor board interface.

Interface number	Main function
E00 or F11	Analog input channel 0 or differential forward 11 port
E1 or F12	Analog input channel 1 or differential forward 12 ports
E2 or F13	Analog input channel 2 or differential forward 13 ports
E3 or F14	Analog input channel 3 or differential forward 14 ports
E4 or F15	Analog input channel 4 or differential forward 15 ports
E5	Analog input channel 5
E6	Analog input channel 6
E7	Analog input channel 7

**Table 2:** Collected data and mode judgment results.

Grid numbering	Data collected by sensor nodes (mV)										Damage mode
	1	2	3	4	5	6	7	8	9	10	
1	14	10	13	12	13	13	11	9	−2	0	1
2	13	8	14	11	12	13	13	13	0	1	2
3	12	7	13	9	9	12	13	14	0	6	3
4	0	−2	1	2	12	11	10	15	10	8	4
5	0	0	1	1	11	12	12	10	9	8	5
6	1	0	1	1	10	12	12	13	8	8	6
7	0	−2	0	0	−2	1	1	14	12	8	7
8	0	−2	0	0	−2	1	1	2	11	8	8
9	−2	−2	−2	−2	0	1	1	1	8	8	9

**Table 3:** Comparison results of monitoring accuracy of sports injury data between two systems.

Grid number	Damage mode	Traditional system (%)	This article system (%)
1	1	50	89
2	2	23	90
3	3	45	92
4	4	61	95
5	5	59	96
6	6	72	93
7	7	81	94
8	8	65	96
9	9	67	91

## Data Availability

The data used to support the findings of this study are available from the corresponding author upon request.
